# Feature Recognition and Style Transfer of Painting Image Using Lightweight Deep Learning

**DOI:** 10.1155/2022/1478371

**Published:** 2022-07-05

**Authors:** Yuanyuan Tan

**Affiliations:** College of Art and Design, Hunan First Normal University, Changsha 410205, China

## Abstract

This work aims to improve the feature recognition efficiency of painting images, optimize the style transfer effect of painting images, and save the cost of computer work. First, the theoretical knowledge of painting image recognition and painting style transfer is discussed. Then, lightweight deep learning techniques and their application principles are introduced. Finally, faster convolutional neural network (Faster-CNN) image feature recognition and style transfer models are designed based on a lightweight deep learning model. The model performance is comprehensively evaluated. The research results show that the designed Faster-CNN model has the highest average recognition efficiency of about 28 ms and the lowest of 17.5 ms in terms of feature recognition of painting images. The accuracy of the Faster-CNN model for image feature recognition is about 97% at the highest and 95% at the lowest. Finally, the designed Faster-CNN model can perform style recognition transfer on a variety of painting images. In terms of style recognition transfer efficiency, the highest recognition transfer rate of the designed Faster-CNN model is about 79%, and the lowest is about 77%. This work not only provides an important technical reference for feature recognition and style transfer of painting images but also contributes to the development of lightweight deep learning techniques.

## 1. Introduction

With the development of network technology, computer technology has become the mainstay of various industries in the development of human society. As relatively comprehensive computer technology, machine learning, including deep learning technology, is also the focus of current social research. Therefore, deep learning technology has been comprehensively developed in many industries [1]. As an important project in the field of art, painting images have become a research hotspot for image feature recognition and style transfer [2]. The innovation lies in the feature recognition and style transfer research of painting images through lightweight deep learning technology. Although this identification and migration work is not yet mature, many studies have provided technical support.

Shen et al. [3] pointed out that, with the development of computer technology, professional computer technology has gradually emerged and played an important role in the field of image recognition. Therefore, image recognition technology based on deep learning has been developed to improve image recognition accuracy and has become one of the main technologies that people apply in real life. However, the current network image recognition technology has many shortcomings, including high computational cost, large storage capacity, and unstable algorithms. Maqsood et al. [4] proposed a lightweight image recognition and segmentation technique using depthwise separable convolutions. Its main idea is to realize image distribution recognition through image segmentation. Then, the technique fuses the distributed features of the image. Finally, the comprehensive features of the images are aggregated to improve image recognition efficiency. Ibrahim et al. [5] proposed an improved backpropagation neural network (BPNN) for image feature recognition and learning algorithm and gave the adjustment method of momentum coefficient and learning rate. After research, the accuracy of each index output by the neural network has been significantly improved, and the average recognition accuracy of the microphone image features has reached 92.7%. The recognition speed also meets the requirements of online real-time detection. Hollandi et al. [6] proposed a concept of image segmentation to realize the conversion of different styles of images. Through image segmentation, the application of image transfer algorithms and style transfer was realized. This method can make the image transfer style according to the need to perform the synchronous transfer of different parts, increase the accuracy of image style transfer, and realize the lightweight optimization of image style transfer. Currently, computers are used to realize image feature recognition and style transfer are relatively advanced methods. However, the implementation of this technology is too much work. Therefore, it is light-provisioned to achieve lightweight technology. Therefore, lightweight deep learning technology is used to realize feature recognition and style transfer of painting images, which is a better method at present.

To sum up, first, the theoretical knowledge of painting image recognition and style transfer is discussed. Then, lightweight deep learning techniques and their application principles are introduced. Finally, through a lightweight deep learning model, faster-convolutional neural network (Faster-CNN) image feature recognition and style transfer models are designed. The innovation is that it can change the traditional method of painting image feature recognition and style transfer and realize the accurate image feature recognition and painting style transfer process under the lightweight deep learning technology. This study not only provides a technical reference for feature recognition and style transfer of painting images but also contributes to the development of lightweight deep learning techniques.

## 2. Research Theories and Methods

### 2.1. Feature Recognition of Painting Images

At present, all kinds of science and technology have become the main support point of human life. Therefore, the use of science and technology to transform various fields has become the main driving force for human development [7]. As a common form of information transmission in human life, image acquisition has become one of the mainstream technologies in society. The information image contained in the image can fill some of the shortcomings of human information acquisition technology. Therefore, the importance of image information is self-evident. However, how to accurately obtain the information in the image through science and technology is the main problem at present [8].

As an art form that plays an important role in human development, painting carries the development history of a nation. Additionally, it also reflects the life characteristics of a nation. Therefore, painting is an important part of a national culture [9]. It not only reflects the cultural appearance and aesthetic characteristics of the nation in various forms but also reflects the development process of the nation. It is a unique and important way for human beings to observe and express the world [10]. In the long history of human development, countless paintings and images have been produced. The study of these paintings can not only have a more comprehensive understanding of the development process but also comprehensively understand the development of human civilization and promote the development of human beings [11].

In the long-term process of painting feature recognition, human beings rely the most on digital image recognition technology. This technique can only identify a single feature of an image by its face. As human beings continue to generate comprehensive needs for image features, a single image feature recognition method can no longer meet people's needs [12]. People need more comprehensive image feature recognition technology to explore more comprehensive image information and obtain various information contained in images more comprehensively and accurately [13]. As a relatively mature machine learning technology, deep learning technology can comprehensively extract and recognize image features through deep learning and computational analysis and has become the main technology in image recognition [14]. The specific principles of image recognition technology under different technologies are shown in Figure 1.

In Figure 1, the traditional image recognition technology that relies on digital technology can only recognize a single image feature and cannot recognize other elements in a complex image. Deep learning technology can recognize all the features in the image in all aspects and can comprehensively analyze the complex elements in the image, which has made an important contribution to the development of human image recognition [15].

### 2.2. Image Style Transfer

Style transfer is the transformation of an ordinary image into another style. Transfer generally includes two types of methods, namely, simulation-based rendering techniques and learning-based rendering techniques. The technology based on simulation drawing focuses on imitating the real painting process and is more suitable for hand-drawn paintings, such as oil paintings or sketches [16]. Learning-based rendering techniques focus on learning the texture features of images and are used in a wider range. The art style is a relatively stable overall artistic feature presented by the interaction between the artist's creative personality and the language and situation of the artwork. In the history of human painting, each drawing may present a different artistic style. As nonart majors, everyone has their own opinions on style. How to change the style of one image to another is even more difficult to define. For programmers, especially machine learning programmers, how to turn an inexplicable thing into an executable program is a problem that plagues many researchers in image style transfer [17]. The specific principle of image style transfer is shown in Figure 2.

Figure 2(a) is the style transfer for fruit painting; Figure 2(b) is the style transfer for train images. Different styles will change the basic form of the image, and the field to which the basic style of the image is applied will also change. Therefore, to meet people's needs for different styles of images, the original images are style-transferred to make certain changes according to different style standards to meet different application needs. In the long-term development of deep learning technology, through image recognition and image feature extraction, according to the image style template, the technology of image-oriented style transfer has become the current mainstream technology after long-term development. Therefore, the study of image style transfer through deep learning technology can not only meet the needs of human beings for different styles of images but also comprehensively promote the development and application of deep learning technology [18].

### 2.3. Lightweight Deep Learning Technology

Since the end of the twentieth century, artificial neural network (ANN) technology has been greatly developed due to its unique properties. The design of this technology mainly refers to the human nervous system. That is, a neural network layer with different properties is constructed through many neurons. Then, a huge neural network system is built from these network layers. Finally, the constructed neural network system can simulate the analysis properties of the human neural network system to a great extent. Therefore, the style exhibited by ANN when dealing with tasks is very human-friendly [19]. The basic structure of neural network technology includes input, hidden, and output layers. Among them, the hidden layer is the main computing level of neural network technology, and its network structure is very deep.

Among neural network technologies, convolutional neural network (CNN) technology is a neural network that focuses on processing images. The technology has evolved considerably since its original design. Therefore, CNN has made an important contribution to humans in the process of processing image information. However, the computationally heavy process of this technology also limits its application in various fields. Therefore, reducing the computational cost of CNN and shortening the computation time, comprehensively optimizing the technology, and highlighting its contribution to image recognition technology are the main research purposes in the current image recognition field [20].

CNN is a kind of neural network that imitates the visual structure of biology, and it is an efficient recognition algorithm. This recognition algorithm mainly includes convolutional, pooling, and fully connected layers. The convolution operation of the convolutional layer is one of the main operations of CNN. The convolution calculation of continuous functions is shown as follows:

(1) $$\begin{array}{c} s\left(t\right)=\int x\left(a\right)w\left(t-a\right)da. \end{array}$$

In (1), **x** and **w** represent integrable functions; **a** and **t** represent different computational elements; **d** represents the convolution operation. The convolution calculation of discrete functions is shown as follows:

(2) $$\begin{array}{c} s\left(n\right)=\sum_{m}r\left(m\right)v\left(n-m\right). \end{array}$$

In (2), **r** and **v** denote discrete functions; **m** and **n** denote calculation elements [21]. In computer vision tasks, convolution can be regarded as a filtering operation. Usually, a two-dimensional image is used as input data. A two-dimensional discrete convolution is used during convolution as follows:

(3) $$\begin{array}{c} I\left(x,y\right)*k\left(x,y\right)=\sum_{s=0}^{m}\sum_{t=0}^{n}k\left(s,t\right)I\left(x-s,y-t\right). \end{array}$$

In (3), **I** represents the output feature; **k** represents the convolution kernel; **m** and **n** represent the dimensions of the convolution kernel; **x** and **y** represent the point of feature output; **s** and **t** represent the feature extraction point. The functions of the pooling and the fully connected layer are to pool the image and output the result, respectively. The computation of the CNN model includes forward and backward propagation. Forward propagation is a series of computing operations such as image recognition and image feature extraction through input data, and the results are integrated and output. Backpropagation refers to the input of the calculation results to calculate the error as the basic reference information for model optimization. Through continuous iterative training and updating, the parameters learned by the network are optimized, and the training is terminated when the artificially set conditions are reached [22]. Among them, the calculation process of backpropagation is to forward the input sample (**x**, **y**) to calculate the output value of **L**_1_, **L**_2_,…, **L**_**n**_ and the error of the output layer as follows:

(4) $$\begin{array}{c} \delta_{i}^{\left(n_{i}\right)}=-\left(y-a^{\left(n_{i}\right)}\right)\cdot f^{\prime }\left(z_{i}^{\left(n_{i}\right)}\right). \end{array}$$

The error calculation of each layer is shown as follows:

(5) $$\begin{array}{c} \delta^{\left(l\right)}=\left({\left(W^{\left(l\right)}\right)}^{T}\delta^{\left(l+1\right)}\right)f^{\prime }\left(z^{\left(l\right)}\right). \end{array}$$

The partial derivatives of weights and biases are calculated as follows:

(6) $$\begin{array}{c} \nabla_{w^{\left(l\right)}}J\left(W,b;x,y\right)=\delta^{\left(l+1\right)}{\left(a^{\left(l\right)}\right)}^{T}, \end{array}$$

(7) $$\begin{array}{c} \nabla_{b^{\left(l\right)}}J\left(W,b;x,y\right)=\delta^{\left(l+1\right)}. \end{array}$$

The updated weight parameters are as follows:

(8) $$\begin{array}{c} W^{\prime }=W^{l}-\mu \nabla_{W^{\left(j\right)}}J\left(W,b;x,y\right), \end{array}$$

(9) $$\begin{array}{c} b^{\prime }=b^{l}-\mu \nabla_{b^{\left(i\right)}}J\left(W,b;x,y\right). \end{array}$$

*δ* represents the difference between the true and the predicted value of the network; **W** represents the weight; **b** represents the bias of the neuron; **z** represents the input of the neuron; **a** represents the output of the neuron; **f**′(**z**^(*l*)^) represents the activation function; *μ* represents the learning rate; *l* represents the level of neurons; **i** represents neurons; **T** represents a constant. The loss function of a sample is calculated as follows:

(10) $$\begin{array}{c} J\left(W,b;x,y\right)=\frac{1}{2}{\left\|y-h_{W^{\prime },b}\left(x\right)\right\|}^{2}. \end{array}$$

The staggered computation of neurons is shown as follows:

(11) $$\begin{array}{c} \delta_{i}^{\left(n_{l}\right)}=\frac{\partial }{\partial z_{i}^{\left(n_{l}\right)}}\frac{1}{2}{\left\|y-h_{w,b}\left(x\right)\right\|}^{2} \end{array}$$

(12) $$\begin{array}{c} h_{w,b}\left(x\right)=a_{i}^{\left(n_{l}\right)}=f\left(z_{i}^{\left(n_{l}\right)}\right). \end{array}$$

To reduce storage space and computational consumption, the CNN model v is compressed. Here, the compression processing method is a matrix decomposition method. This method incorporates the singular value decomposition (SVD) algorithm. The SVD algorithm is a very important model compression method. Its connotation is to represent the original matrix by extracting key features; that is, a complex matrix is approximated by multiplying several small matrices representing key features in the original matrix [23]. SVD is an algorithm widely used in the field of machine learning. It can be used not only for feature decomposition in dimensionality reduction algorithms, but also for recommendation systems and natural language processing. It is the cornerstone of many machine learning algorithms. As a very basic algorithm, SVD has its presence in many machine learning algorithms. In the current era of big data, SVD has a wide range of applications due to its parallelization. The disadvantage of SVD is that the decomposed matrix is not interpretable, but this disadvantage does not affect its use. Singular value decomposition is an algorithm that can be applied to any matrix decomposition; for example, let the data input to the fully connected layer be of size **u** × **v** and the weight matrix be *W*. The calculation of the output data of the fully connected layer is shown as follows:

(13) $$\begin{array}{c} y=W_{x}. \end{array}$$

**W** is used to perform SVD, and the decomposition of **W** is replaced by the first **t** important eigenvalues after decomposition as follows:

(14) $$\begin{array}{c} W=U\sum V^{T}\approx U\sum_{t}V^{T}. \end{array}$$

**U** represents a **u** × **t**-dimensional orthogonal matrix; ∑ represents a diagonal matrix; **V** represents a **v** × **t**-dimensional orthogonal matrix. Therefore, the representation of SVD is as follows:

(15) $$\begin{array}{c} y=Wx\approx U\cdot \left(\sum_{t}V^{T}\right)\cdot x=U\cdot z. \end{array}$$

The SVD algorithm can decompose the CNN technology, which greatly reduces the computational load of the network. This method is not only simple but also achieves better results. Another method is the low-rank decomposition (LRD) algorithm. This algorithm is an optimization algorithm for the SVD. The SVD algorithm cannot solve the simpler computational operations of images, and the LRD algorithm can solve this problem well [24]. The definition of its output feature map is shown as follows:

(16) $$\begin{array}{c} F_{n}\left(x,y\right)=\sum_{i=1}^{C}\sum_{x^{\prime }=1}^{X}\sum_{y^{\prime }=1}^{Y}Z^{c}\left(x^{\prime },y^{\prime }\right)W_{n}^{c}\left(x-x^{\prime },y-y^{\prime }\right). \end{array}$$

**W** represents the channel, **n** represents the filter, and **C** represents the channel's position. The main purpose is to find an approximation of **W**, $\hat{W}$ as follows:

(17) $$\begin{array}{c} {\hat{W}}_{n}^{c}=\sum_{k=1}^{K}H_{n}^{k}{\left(V_{k}^{c}\right)}^{T}. \end{array}$$

**K** represents the hyperparameter that controls the rank; **H** represents the horizontal filter; **V** is the vertical filter. However, LRD also has certain disadvantages. That is, although LRD has achieved good results for model compression and acceleration, the implementation of this method is not easy. There are decomposition operations with high computational costs. Since different layers contain different information, it is not possible to use a global variable to implement LRD, and it is necessary to perform low-rank approximation (LRA) layer by layer. Moreover, after being decomposed, a lot of fine-tuning training is required to make the network converge to achieve the optimal effect [25].

### 2.4. Optimized Lightweight Faster-CNN Algorithm

Machine learning has developed for a long time since its inception, and it has accumulated many shortcomings. Traditional machine learning techniques require continuous design by humans to gradually improve their own learning process. Therefore, in the calculation process, its dependence is particularly large, and the basic technical ability of the operator is relatively high. The development of machine learning has also been greatly limited. Meanwhile, the algorithm's accuracy for image recognition is very low, and it cannot quickly achieve accurate image recognition [26]. Among them, the most important is that the traditional machine learning technology cannot accurately identify various factors in the image, which usually causes large errors in the application. The most serious is that machine learning cannot classify the main part and background part of the image and cannot identify the main information contained in the image [27]. The optimized deep learning technology solves the shortcomings of traditional machine learning technology in image recognition. If deep learning image recognition technology needs to be pushed to a wider field, it is necessary to optimize its calculation process to reduce its computational cost and improve its computational efficiency. Therefore, by optimizing the CNN technology and generating the Faster-CNN model, the model calculation process is simpler, and the calculation effect is also improved to a certain extent. The basic idea of the designed lightweight Faster-CNN model is shown in Figure 3.

In Figure 3, when the Faster-CNN model is used for image feature recognition, it can not only greatly reduce the process of image feature recognition and improve the efficiency of image feature recognition but also optimize the recognition effect of the model and better help people to complete the style transfer of painting images. The approach adopted when optimizing the Faster-CNN model is the region proposal network. It adjusts and optimizes the image recognition area of the Faster-CNN model through anchor points as follows:

(18) $$\begin{array}{c} x=w_{a}t_{x}+x_{a}, \end{array}$$

(19) $$\begin{array}{c} y=h_{a}t_{y}+y_{a}, \end{array}$$

(20) $$\begin{array}{c} w=w_{a}\left(t_{w}\right), \end{array}$$

(21) $$\begin{array}{c} h=h_{a}\left(t_{h}\right). \end{array}$$

**x**_**a**_, **y**_**a**_, **w**_**a**_, and **h**_**a**_, respectively, represent the abscissa and ordinate of the center point of the anchor point and the width and height of the anchor point. **x**, **y**, **w**, and **h** represent the horizontal and vertical coordinates of the center selected by the model, as well as the selected width and height, respectively. **t** represents the corrected value.

### 2.5. Description of Study Data

Public datasets are used to train the model comprehensively. The comprehensive performance of the model is evaluated. Here, the adopted dataset includes the Mixed National Institute of Standards and Technology (MNIST) dataset. The MNIST dataset is one of the most popular deep learning datasets. It is a dataset of handwritten digits containing a training set of 60,000 examples and a test set of 10,000 examples. This is a great database for trying out learning techniques and deeply identifying patterns in real data that can spend minimal time and effort in data preprocessing. The open images dataset is a dataset of nearly nine million images of uniform resource locations (URLs). These images span thousands of class image-level label bounds and are annotated. The dataset contains a training set of 9,011,219 images, a validation set of 41,260 images, and a test set of 125,436 images. The Canadian Institute For Advanced Research-10 (CIFAR-10) dataset is another dataset for image classification. It consists of 60,000 images of 10 classes (each class is represented as a row in the image above). There are 50,000 training and 10,000 test images in total. The dataset is divided into six parts: five training batches and one testing batch. Each batch has 10,000 images. The ImageNet dataset is an image dataset organized based on the WordNet hierarchy. WordNet contains about 100,000 phrases, and ImageNet provides an average of about 1000 images to illustrate each phrase. The total number of images is about 1,500,000. Each image has multiple bounding boxes and corresponding class labels.

## 3. Drawing Image Feature Recognition and Evaluation of Style Transfer

### 3.1. Identification and Evaluation of Image Features

To improve the computing efficiency and save computing costs and storage space of the deep learning technology, the lightweight deep learning model can be optimized to meet the demand for image feature recognition using the lightweight deep learning model. The average rate of image recognition of the designed model is shown in Figure 4.

In Figure 4, in the image recognition rate evaluation of the lightweight deep learning model, the designed Faster-CNN model has little difference between the image recognition rates of the SVD and LRD algorithms. The designed Faster-CNN model has the highest average recognition time of about 28 ms in the four datasets, and the lowest is about 17.5 ms. The average image recognition time of the SVD algorithm is around 31 ms at the highest and around 18 ms at the lowest. The average image recognition time of the LRD algorithm is around 30 ms at the highest and around 20 ms at the lowest. The designed model still has advantages over SVD and LRD algorithms. While focusing on the recognition efficiency of the model, it is generally necessary to evaluate the accuracy of the model to determine its comprehensive advantages. The results of the image recognition accuracy evaluation of the model are shown in Figure 5.

In Figure 5, the image recognition accuracy of the designed Faster-CNN model is around 97% at the highest and around 95% at the lowest. The image recognition rate of the SVD algorithm is around 97% at the highest and around 93% at the lowest. The image recognition rate of LRD is around 95% at the highest and around 92% at the lowest. The Faster-CNN model has great advantages in image recognition accuracy.

### 3.2. Transfer Evaluation of Painting Image Styles

With the development of science and technology, the style transfer of painting images has become a technology that can be generally realized. However, its efficiency and accuracy also need to be improved to a certain extent to achieve an efficient transfer of painting image styles. The results of images being transferred with different styles are shown in Figure 6.

In Figure 6, the Faster-CNN model can identify and transfer styles of various painting images, so that the styles of the images are transformed into images of other styles. The designed model also has great advantages in the transfer efficiency of image style recognition. The evaluation results of the transfer efficiency of painting image recognition of the Faster-CNN model are shown in Figure 7.

In Figure 7, the Faster-CNN model has a great advantage in transferring painting image style recognition. Among the five groups of image style recognition migration, the recognition migration rate of the Faster-CNN model is the highest at around 79% and the lowest at around 77%. The SVD algorithm recognizes that the highest mobility rate is around 74%, and the lowest is around 71%. The LRD algorithm recognizes that the highest mobility is around 74%, and the lowest is around 70%. The designed Faster-CNN model still has a strong advantage in the style transfer of painting images.

## 4. Conclusion

With the development of science and technology, deep learning technology has become a relatively advanced computer technology. The lightweight deep learning model has been greatly optimized in terms of storage and computation based on inheriting the deep learning model technology. First, the theoretical knowledge of painting image recognition and style transfer is discussed. Then, lightweight deep learning techniques and their application principles are introduced. Finally, based on the lightweight deep learning model, Faster-CNN image feature recognition and style transfer models are designed. Model performance is comprehensively evaluated. Studies showed that the designed Faster-CNN model has the highest average recognition time of about 28 ms and the lowest of about 17.5 ms in feature recognition of painting images. The accuracy of the Faster-CNN model for image feature recognition is about 97% at the highest and 95% at the lowest. Finally, the designed Faster-CNN model can perform style recognition transfer on various painting images. In terms of style recognition transfer efficiency, the highest recognition transfer rate of the designed Faster-CNN model is about 79%, and the lowest is about 77%. The innovation lies in transforming traditional image feature recognition and style transfer methods and realizing painting image feature recognition and style transfer technology under the lightweight deep learning technology. This study designs a model with painting image recognition and style transfer, but the shortcomings of the model have not been comprehensively studied. Therefore, future research will strengthen the development of model defects to optimize and improve the model performance continuously.

## Figures and Tables

**Figure 1:** The specific principles of image recognition technology under different technologies. (a) Traditional image recognition. (b) Deep learning technology image recognition.

**Figure 2:** The transfer principle of image style. (a) Fruit. (b) Training.

**Figure 3:** The basic idea of the lightweight Faster-CNN model.

**Figure 4:** The lightweight deep learning model for image recognition rate. (a) MNIST dataset. (b) Open images dataset. (c) CIFAR-10 dataset. (d) ImageNet dataset.

**Figure 5:** The image recognition accuracy of lightweight deep learning models. (a) MNIST dataset. (b) Open images dataset. (c) CIFAR-10 dataset. (d) ImageNet dataset.

**Figure 6:** The transfer results of the recognition style of the painting image of the lightweight deep learning model. (a) Stone tools. (b) Architecture and landscape. (c) Landscape. (d) Pure architecture. Image source is the network.

**Figure 7:** Evaluation of transfer efficiency for style recognition in painting images.

## Data Availability

The data used to support the findings of this study are included within the article.
